# ZFP36 Inhibits Tumor Progression of Human Prostate Cancer by Targeting CDK6 and Oxidative Stress

This article has been retracted.

**DOI:** 10.1155/2022/3611540

**Published:** 2022-09-06

**Authors:** Dongbo Yuan, Yinyi Fang, Weiming Chen, Kehua Jiang, Guohua Zhu, Wei Wang, Wei Zhang, Ganhua You, Zhenyu Jia, Jianguo Zhu

**Affiliations:** ^1^Medical College of Guizhou University, Guiyang, Guizhou Province 550025, China; ^2^Department of Urology, Guizhou Provincial People's Hospital, The Affiliated Hospital of Guizhou Medical University, Guiyang, Guizhou Province 550002, China; ^3^The Second People's Hospital of Guizhou Province, Guiyang, Guizhou Province 550000, China; ^4^Department of Plant and Botany Sciences, University of California of Riverside, Riverside, CA 92521, USA

## Abstract

**Background:**

The expression of ZFP36 in previous study was reduced in prostate cancer (PCa) tissues as compared to benign prostate tissues, indicating the potential of ZFP36 as an auxiliary marker for PCa. Further evaluation was conducted in clinical samples for in vitro and in vivo experiments, to prove the potential possibility that ZFP36 dysregulation participated in the malignant phenotype of PCa, to determine its potential mechanism for tumor regulation, and to provide a new theoretical basis for gene therapy of PCa.

**Methods:**

First, the expression of ZFP36 in prostate tissue and PCa tissue was explored, and the relationship between ZFP36 and clinical features of PCa patients was illustrated. Subsequently, the impact of ZFP36 on the biology of PCa cells and relevant downstream pathways of ZFP36's biological impact on PCa were elucidated. Finally, whether oxidative stress mediated the regulation of ZFP36 in PCa was verified by the determination of oxidative stress-related indicators and bioinformatics analysis.

**Results:**

The downregulation of ZFP36 in PCa tissue had a positive correlation with high Gleason scores, advanced pathological stage, and biochemical recurrence. ZFP36 was identified as an independent prognostic factor for PCa patients' BCR-free survival (*P* = 0.022) by survival analysis. Following a subsequent experiment of function gain and loss, ZFP36 inhibited the proliferation, invasion, and migration in DU145 and 22RV1 cells and inhibits tumor growth in the mouse model. Additionally, high-throughput sequencing screened out CDK6 as the downstream target gene of ZFP36. Western blot/Q-PCR demonstrated that overexpression of ZFP36 could reduce the expression of CDK6 at both cellular and animal levels, and the dual-luciferase experiment and RIP experiment proved that CDK6 was the downstream target of ZFP36, indicating that CDK6 was a downstream target of ZFP36, which mediated tumor cell growth by blocking cell cycle at the G1 stage. Furthermore, ZFP36 inhibited oxidative stress in PCa cells.

**Conclusions:**

In PCa, ZFP36 might be a tumor suppressor that regulated growth, invasion, and migration of PCa cells. The lately discovered ZFP36-CDK6 axis demonstrated the molecular mechanism of PCa progression to a certain extent which might act as a new possible therapeutic target of PCa therapy.

## 1. Introduction

The proteins controlling multiple cellular phenotypes of proliferation, differentiation, apoptosis, cell invasion, cell cycle, and angiogenesis, once with abnormal expression, can cause the exacerbation of cancer initiation and progression [1]. The influential factor for such protein synthesis is positively correlated with the cytoplasmic concentrations of the corresponding mRNAs and consequently depends on the kinetics of mRNA synthesis and degradation. It has been recognized that 2 in 3 of the variation in protein abundance of mammalian cells are accounted for the mechanism of posttranscription [2]. Posttranscriptional regulation is critical for biological processes and pathologies [3–5]. Both miRNAs and RNA-binding proteins (RBPs) have been identified as the principal decisive factors for posttranscriptional control [6]. As noncoding protein RNAs, miRNAs are known as small as 22 nt, and they negatively mediate the expression of genes on posttranscription, cleavage the target mRNAs by primarily binding to the 3′-untranslated regions (UTRs) of targets, and inhibit translation process when complementary sites are insufficient [7]. Through participating in the whole processes of posttranscriptional regulation, the RBPs determine cell fate and function of transcripts and ensure cellular homeostasis. These proteins can create frequent dynamic interactions with coding and noncoding RNAs and additional proteins, thereby mediating RNA shearing, translation, stability, and degradation [8, 9]. In different cancer types, RBPs are dysregulated, thereby affecting the expression of both oncoproteins and tumor suppressor proteins as well as corresponding functions. Therefore, investigation of interrelationship between RBPs and the corresponding targets of cancer-associated RNA can benefit a lot in tumor biology recognition and it may identify potential targets for cancer management.

The best phenotype of RNA-binding protein is Tristetraprolin (TTP) and recognized as ZFP36, G0S24, Nup475, and TIS11. The property of the TTP family includes three cysteine (C) residues and one histidine (H) residues. ZFP36 or TTP, ZFP36L1, and ZFP36L2 are the human members in the family [10]. The TTP family binds to AREs with a specific sequence and structure via the zinc finger domain. Meanwhile, it can catalyze poly (a) tail removal, as a result of mRNA attenuation. It has been revealed by genomic analysis that AREs present in at least 11% of human genes, and all ten molecular mechanisms defined as “cancer hallmarks” include ARE-containing genes [11, 12]. AREs can bind to proteins, namely, TTPs, and they ensure the stability of transcripts or the direct damage of them [13]. As commonly seen in various mRNAs encoding cancer-related proteins, the expression and/or activity of ARE-BPs is associated with tumorigenesis or progression of tumors. Some studies have reported that model mice with TTP knockout perform normal behaviors at birth, but develop a systemic inflammatory syndrome within 2-3 weeks, including cachexia, arthritis, myeloid hyperplasia, and autoimmune diseases [14]. TTP can directly mediate zinc finger E-box-binding homeobox 1 (ZEB1), SRY gene 9 (SOX9), EMT regulators, and colon cancer metastasis-associated 1 (MACC1); all of these factors are downregulated in colorectal cancer [15]. TTPs play an important role as tumor suppressors; it has been found that MYC oncoprotein can directly inhibit the transcription of TTP; the inhibition of which may be a feature of MYC-involved malignancies [16]. Taken together, the previously described studies have demonstrated the intimate and complicated relationship between ARE-BPs and cell growth, apoptosis, angiogenesis, and the development stages of tumors.

Prostate cancer (PCa) ranks the fifth of malignant tumors in global tumor incidence and the second mortal malignant tumor in the world (after lung cancer) [17–19]. Despite multiple mRNAs encoding tumorigenic products being possibly mediated by AREBPs, dysregulation of ARE-BP expression and/or activity in PCa development remains unknown. Our previous study indicated a marked decrease of ZFP36 protein expression in PCa tissues versus non-PCa tissues, which indicated that this protein was involved in PCa progression [20].

To address this issue, we employed a database to analyze ZFP36 expression in PCa. Meanwhile, the association between clinicopathological features and prognosis was also explored. Given that we observed expression of ZFP36 was reduced in many cancers, we predicted that reducing ZFP36 levels might increase the tumorigenic phenotype. To validate this model, experiments were performed at the cell and animal levels. Further, high-throughput sequencing and bioinformatics methods were conducted to determine the specific mechanism by which ZFP36 was involved in tumors. These results would help to provide personalized and precise treatment for PCa patients.

## 2. Materials and Methods

### 2.1. Patient Enrollment and Sample Collection

The experiments of the present study have gained the approval of human study ethics committees at MGH, Boston, MA, and Ministry of Public Health of P.R. China. The recruited patients have signed written informed consent. And the specimens have been collected anonymously as per the ethical and legal laws and regulations.

### 2.2. Cell Preparation

Human PCa cell lines DU145, PC-3, 22RV1, and LNCap were from the American Type 6 Culture Collection. By the addition of 10% fetal bovine serum and relevant agents, the cells were cultured in RPMI 1640 medium (Hyclone, USA). Following cell line resuscitation and characterization, passage culture was performed in the laboratory for around 3 months. Reauthentication was not conducted to the cell lines. Short Tandem Repeat (STR) profiling was employed for detection of misidentification, cross-contamination, and genetically drifted cells. The amplification of 17 STR loci plus amelogenin was conducted using the Promega's PowerPlex® 18D System before being kept in a humidified chamber at 37°C with 5% CO_2_.

### 2.3. Animals

All tests followed guidelines of Laboratory Animal Research of Guangzhou Medical University. Twenty male BALB/c nude mice aged 4~5 weeks were from Guangdong Medical Laboratory Animal Center. They were raised in wire-top, sawdust-bedding cages with five in each. The animal room was isolated and clean, with an air conditioner, and the room temperature was set at 25–26°C, relative humidity around 50%, and photoperiod 12 : 12 h.

### 2.4. Cell Line Construction and Transfection

Virus particles were harvested based on instructions of the SBI packaging protocol of Lenti-Concentin Virus Precipitation Solution (Cat No. LV810A-1). Both cells DU145 and LNCap were infected using the TransDux virus transduction reagent (Cat No. LV850A-1) (SBI, USA). The following isolation used a flow cytometer, and the infected cells were cultured in 96-well plates [21].

### 2.5. qRT-PCR

Expression levels of ZFP36, TGFBR2, LAMC1, CDK6, NKX3-1, PCDH7, PARVA, and KRT14 mRNA in xenograft tumors, clinical PCa tissues, and cell lines were determined via qRT-PCR assays as per procedures of our previous study [22].

### 2.6. Western Blot Analysis

Expression of PCa cell line proteins, xenograft tumors, and PCa tissues was determined using western blot as per procedures of our previous study [22].

### 2.7. Immunohistochemistry

Immunohistochemistry was conducted to examine the expression patterns of MMP9, vimentin, Ki-67, E-cadherin, and caspase-3 proteins and their subcellular locations in subcutaneous tumors of animals. Meanwhile, immunoreactivity score (IRS) of vimentin was obtained based on previously described procedures in our study.

### 2.8. Xenograft Model Construction In Vivo

We subsequently performed tumor formation assay in vivo. After transfection of DU145 or 22RV1 cells with ZFP36, NC lentivectors were trypsinized for suspension in phosphate-buffered saline (PBS). Each nude mouse was subcutaneously injected with the following cells (5 per group): DU145 at a concentration of 1 × 10^6^, 22RV1 at a mixture of 2 × 10^6^ of 10 mg/mL. In a 4-day interval, the tumor sizes were measured when available for measurement. The calculation of tumor volume was as per *V*(mm^3^) = width^2^ (mm^2^) × length (mm)/2. The animals were sacrificed for the experiments on days 36 and 44 for DU145 and 22RV1, respectively. They were fed in accordance with the protocols of Laboratory Animal Research at Guangzhou Medical University [23].

### 2.9. Luciferase Reporter Assay

ZFP36 targeted gene expression in DU145 cells was determined through luciferase reporter assays. Putative complementary site of ZFP36 at CDK6 mRNA 3′-UTR or mutant sequence was cloned into the luciferase reporter vector psiCHECK-2 (Promega, USA). DU145 cells were cotransfected with 50 nM ZFP36 mimic or the negative control and 0.5 *μ*g of psiCHECK-2-ZFP36–3′-UTR-WT or psiCHECK-2-ZFP36–3′-UTR-MUT. Following 48 h, cells were harvested for analysis using Dual-Luciferase Reporter Assay System (Promega, USA). Simultaneously, the GloMax fluorescence reader (Promega, USA) was employed to generate firefly and renilla luciferase signals, and the latter was normalized the firefly luciferase signals [24].

### 2.10. Transwell Assays

To further determine invasion and migration of cells, Transwell and scratch wound-healing motility was performed following procedures described previously.

### 2.11. RNA Immunoprecipitation Assay

Cells were scraped from the Petri dish and collected into a 1.5 mL tube, resuspended the magnetic beads, suck 50 *μ*L of the resuspended magnetic bead suspension into each Eppendorf tube, resuspend the magnetic beads with 100 *μ*L of RIP wash buffer, add about 5 *μ*g of the corresponding antibody into each sample, put the Eppendorf tube on the magnetic rack, remove the supernatant, add RIP immunoprediction buffer into each tube, take 50 *μ*L of supernatant as input for RNA, and put the remaining supernatant into the magnetic bead antibody complex. The total volume was 1 mL and incubated at 4°C for 3. Add 500 *μ*L RIP wash buffer, place the Eppendorf tube on the magnetic frame after vortex vibration, discard the supernatant, and repeat cleaning 6 times; after rinsing, resuspend the magnetic beads with 100 *μ*L RIP immunoprediction buffer, take 20 *μ*L magnetic beads for each group, add loading buffer to cook the sample, centrifuge at 12000 rpm/min and 4°C for 3 min, and do western blot, and the rest is used to extract RNA.

### 2.12. Apoptosis Assay

Apoptosis of the cells was ultimately examined utilizing the APC-conjugated Annexin V Kit (BD Biosciences, USA) and 7-aminoactinomycin D (Multisciences, China) as per the procedures described in our previous studies.

### 2.13. Enzyme-Linked Immunosorbent Assay (ELISA)

ELISA was conducted to detect SOD, MDA, and ROS of DU145 cell as per instructions of use. Briefly, ELISA kits were equilibrated at room temperature; 50 *μ*L of standard solution and sample was supplied to the sample plates. After being added with 100 *μ*L detection antibody, the well plate was sealed with sealing film and cultured at 37°C for 60 min. 50 *μ*L substrate was provided to each well and incubated in the dark for 15 min. After incubation, stop solution at 50 *μ*L was supplemented, and the OD values at 450 nm were measured for each well.

### 2.14. Data Download and PPI Network Construction

Data related to prostate cancer and oxidative stress were obtained from the database https://www.ncbi.nlm.nih.gov/geo/query/acc.cgi?acc=GSE119005, and PPI diagram was constructed using STRING (http://string-db.org).

### 2.15. GO Enrichment Analysis

Obtained DEGs were subjected to Gene Ontology (GO) analysis with the help of the R software packages clusterProfiler, enrichplot, and ggplot2. Only pathways with both *P* and *Q* values less than 0.05 were regarded as high enrichment.

### 2.16. Statistical Analysis

SPSS and SAS 9.1 were employed for statistical analysis of the obtained data. Continuous variables were expressed as *X̅*±*s*. Wilcoxon signed-rank tests were employed for statistically analyzing qRT-PCR and western blot. Fisher's exact tests were conducted for all 2 × 2 tables and Pearson *χ*^2^ tests for non-2 × 2 tables. Such tests were carried out by two biostatisticians independently. Kolmogorov-Smirnov (K-S) was conducted to test whether the ZFP36 expression was normally distributed. The interrelationship between ZFP36 expression and clinical pathology features of PCa patients in the Taylor dataset was detected using Mann–Whitney *U* tests and Kruskal-Wallis *H* tests. Survival analysis utilized the Kaplan-Meier method, and Cox regression was conducted for univariate and multivariate analyses, *n* = 3. *P* values less than 0.05 were regarded as significant statistical difference.

## 3. Results

### 3.1. ZFP36 Expression Is Decreased in Human PCa Cells and Tissues

First, ZFP36 mRNA expression in all tumors and corresponding healthy tissues was assessed via TCGA database, implying that ZFP36 mRNA expression of most normal tissues in this database was elevated compared to the corresponding cancer tissues (Figure 1(a)); this also fully demonstrated that ZFP36 played a tumor suppressor role in most tumors. Then, the mRNA expression of ZFP36 was evaluated in PCa and normal tissues in TCGA and Taylor public databases (TCGA contains 498 PCa and 52 normal tissues; Taylor contains 150 PCa and 29 normal tissues). The level of ZFP36 mRNA in TCGA database was increased in the normal prostate tissue as compared with PCa (normal: 13.04 ± 1.35; cancer: 12.49 ± 1.52, *P* = 0.012) (Figure 1(b)), while via Taylor database, the expression of ZFP36 mRNA in normal prostate tissue was lower than that in PCa (normal: 9.03 ± 0.76; cancer: 9.47 ± 0.97, *P* = 0.024) (Figure 1(c)). The results in the two databases were inconsistent, but TCGA database included larger sample size, more convincing, and greater reliability. We further tested the expression level of ZFP36 in healthy prostate epithelial cells (RWPE-1), prostate hyperplastic cells (BPH-1), and four PCa cell lines (LNCap, DU145, 22RV1, and PC3). The findings revealed that ZFP36 in RWPE-1 and BPH-1 were highly expressed, but were downregulated in PCa cell lines (Figure 1(d)). We used DU145 and 22RV1 cells for the next experiment.

### 3.2. Decreased Expression of Zn in Human PCa Tissues

Zinc finger proteins refer to a class of proteins that contain short, self-folding “finger” structures that are stabilized by binding Zn^2+^. Human prostates contain higher levels of zinc than most tissues [25]. Unluckily, cellular metabolic alteration exerts an important role in prostate malignancy and has been greatly neglected. Several important factors including zinc have been identified and involved in PCa progression. We reviewed the previous literature summary as shown in Table 1, and we drew the following conclusions: the zinc concentration in healthy prostate tissues and benign prostatic hyperplasia tissue was markedly higher than that in PCa. The marked reduction of zinc concentration in malignant cells represents the biochemical feature of PCa, which is consistent with our findings above that observed decreased expression of zinc finger proteins in PCa.

### 3.3. The Correlation between ZFP36 Expression and Pathological Features of PCa Patients

Furthermore, we used TCGA and Taylor public databases to analyze the correlation between ZFP36 mRNA expression and PCa patients' clinical features. As shown in Table 2 via TCGA database, ZFP36 mRNA level was negatively correlated with Gleason score (*P* = 0.002), pathological stage (*P* = 0.002), and biochemical recurrence (*P* = 0.003); Taylor database indicated that ZFP36 mRNA expression was negatively correlated with Gleason score (*P* < 0.001), pathological stage (*P* = 0.016), distant metastasis (*P* < 0.001), overall survival rate (*P* < 0.001), and biochemical recurrence (*P* < 0.001). Both suggested that ZFP36 expression had a negative correlation with biological characteristics of malignant prostate tumors.

### 3.4. Decreased mRNA Expression Level of ZFP36 Indicates Poor Prognosis of Clinical PCa Patients

Based on TCGA and Taylor clinical PCa databases, we divided the ZFP36 mRNA expression levels into groups of highly and poorly expressed, respectively, based on median, and analyzed expression level of ZFP36 by Kaplan-Meier survival curve and log-rank tests. TCGA database findings indicated that the ZFP36 high expression group had markedly high survival rates free from postoperative biochemical recurrence and metastasis biochemical recurrence than the ZFP36 low expression group (Figure 1(e), *P* < 0.05); in the Taylor database and the ZFP36 high expression group, the postoperative biochemical recurrence-free survival and metastasis-free survival were markedly higher compared with the ZFP36 low expression group (Figure 1(f), *P* < 0.05), indicating that ZFP36 could suppress cancer in prostate tumors.

### 3.5. The mRNA Expression Level of ZFP36 May Serve as an Independent Indicator for Predicting PCa Patients' Prognosis

Furthermore, we used the COX regression model and analyzed predictive ZFP36 mRNA levels in TCGA database on the risk of postoperative biochemical recurrence in PCa patients. The results of univariate analysis revealed that ZFP36 expression, Gleason score, pathological stage, clinical stage, and positive margins might be important predictors of biochemical recurrence in PCa patients (Table 3). Multivariate analysis suggested that ZFP36 expression, Gleason score, and clinical stage might be independent predictors of biochemical recurrence in PCa patients. Consistent with the above-mentioned Kaplan Meier detection and log-rank methods, ZFP36 expression might be a potential prognostic indicator used in predicting patient survival and biochemical recurrence after PCa surgery, further revealing the clinical significance of ZFP36 for PCa patients. Based on the above results, we will further explain the biological function and potential molecular mechanism of ZFP36 on PCa development through experiments in vitro and in vivo.

### 3.6. ZFP36 Can Mediate Proliferation, Migration, and Invasion of PCa Cells In Vitro

We used lentiviral infection technology to construct ZFP36 overexpression and knockdown DU145 and 22RV1 cell lines and their corresponding blank control (negative control (NC)) and used western blot to detect the overexpression and knockdown efficiency of ZFP36. As shown in Figures 2(a)–2(d), ZFP36 overexpressed DU145 and 22RV1, the protein expression of ZFP36 was markedly elevated compared with the NC group, while following ZFP36 knockdown DU145 and 22RV1, the protein expression of ZFP36 was greatly reduced compared with the NC group, indicating that the cell line was successfully constructed and could be used for the next experiment.

In the DU145 and 22RV1 cell lines overexpressing ZFP36, the corresponding cell function experiments were performed. The cell proliferation test results (CCK-8 assay) indicated that tumor cells were significantly decreased after ZFP36 overexpression versus control, implying that ZFP36 could regulate proliferation of PCa tumor cells (Figures 2(e) and 2(h)); then, we performed cell scratch and cell invasion experiments, indicating that overexpression of ZFP36 could greatly suppress migration and invasion of tumor cells versus control (Figures 2(f), 2(i), 2(g), and 2(j)). In general, ZFP36 overexpression could significantly mediate proliferation, invasion, and migration of tumor cells. However, following the inhibition of DU145 and 22RV1 cell lines by ZFP36, the opposite experimental results were revealed: after ZFP36 inhibition, the number of tumor cells increased significantly, and the migration and invasion capabilities of tumor cells were apparently enhanced.

### 3.7. ZFP36 Can Inhibit PCa Growth In Vivo

In the next step, bilateral armpits of nude mice were injected the constructed ZFP36 stable overexpression cell DU145 and corresponding empty vector control cells to construct xenograft tumor models and to remove the tumors from the nude mice subcutaneously after 48 days to measure the tumor size and weight. The results are shown in Figures 3(a) and 3(b). ZFP36-overexpressed DU145 cells could significantly inhibit subcutaneous tumor growth versus control. We also found that ZFP36 overexpression was consistent in 22RV1 cells (Figures 3(c) and 3(d)); in comparison to the control, overexpressing ZFP36 in 22RV1 markedly inhibited tumor growth of nude mice.

In summary, we carried out in vitro experiments using PCa cell lines implying that ZFP36 could mediate proliferation, invasion, and migration of tumor cells. Meanwhile, in vivo tests have confirmed that ZFP36 inhibited tumor growth. From a cellular perspective, the biological characteristics of ZFP36 were preliminary discovered that might inhibit PCa development.

### 3.8. ZFP36 Regulates Prostate Proliferation, Invasion, and Metastasis

To further understand the molecular biological functions of ZFP36 on PCa, we constructed a DU145-ZFP36-overexpressing PCa subcutaneous xenograft model in nude mice. Tissues were collected and immunohistochemical analysis was conducted, indicating that expression of MMP9, vimentin, and Ki-67 was downregulated after ZFP36 overexpression compared with the control group, and so as E-cadherin protein expression, whereas it had no obvious effect on the activation of caspase-3 (Figure 3(e)). As a zinc- and calcium-dependent protease family, matrix metalloproteinases (MMPs) can target numerous proteins in the extracellular matrix and promote their degradation. The extracellular matrix and base together constitute the first barrier in the process of tumor metastasis. Therefore, the degradation of the extracellular matrix often intimately links to the malignant invasion and metastasis of tumors. Vimentin expression can promote the decomposition of intercellular junction proteins and reduce the adhesion between epithelial cells. Vimentin's activation of tumor cell microfilaments and tubulin can improve the deformation and infiltration capacity of epithelial cells. Ki67 is a nuclear antigen that exists in proliferating cells. Its expression and function are linked to chromatin and related to cell mitosis, so it is an extensively applied proliferating cell marker. E-cadherin is an important part of maintaining normal epithelial cell morphology and cell tissue integrity. It can inhibit tumor cell metastasis and invasion and affect tumor growth and proliferation. When E-cadherin protein expression is downregulated, cells lose their ability to adhere to each other; the tumor cells detach from its original site and then metastasize to lymph nodes or far away. Caspase-3 is a protease and well recognized as the most essential terminal splicing enzyme during apoptosis. Meanwhile, it can regulate CTL cell killing mechanism. Our research results suggest that overexpression of ZFP36 can reduce the expression of MMP9, vimentin, and Ki-67 and promote the expression of E-cadherin, thereby mediating various tumor cell processes, which conforms to our above-mentioned cell function experiments. However, it has no obvious effect on the activation of caspase-3, indicating that it may have no effect on tumor cell apoptosis.

### 3.9. Pathways Related to ZFP36 in PCa

DEGs between ZFP36 inhibition and control DU145 were determined by NGS RNA technique to clarify potential mechanism of ZFP36 in the progression of PCa. Consequently, in DU145 cells inhibited by ZFP36, based on |logFC| > 1 of the differential gene, we identified a total of 341 dysregulated genes with 229 upregulated and 112 downregulated (Figure 4(a)). The KEGG enrichment analysis shown in Figure 4(b) shows that the target genes regulated by ZFP36 are mainly related to PI3K-Akt signaling pathway, circadian rhythm, cell matrix adhesion, HIF-1 and Rap1 signaling pathways, and cancer pathway. Meanwhile, GO analysis (Figure 4(c)) revealed that the protein altered by ZFP36 significantly controls multiple biological processes directly related to cancer, namely, cell growth, regulation of cell growth, extracellular matrix tissue, and extracellular structural tissue, involving several processes of cell viability and growth, and there is evidence indicating that abnormal regulation of cell viability and growth components may be the cause of tumor formation. Generally, ZFP36 candidate target is associated with a wide range of biological functions related to PCa.

### 3.10. CDK6 Is the Direct Target of ZFP36

According to |logFC| > 1 of the differential gene in the DU145-KO-ZFP36 sequencing results, the oncogenes in the KEGG database or the biochemical recurrence meaningful genes in the comprehensive Taylor database were jointly screened for related genes downstream of ZFP36 (TGFBR2, LAMC1, CDK6, NKX3-1, PCDH7, PARVA, and KRT14), but only CDK6 screened for all three of them presented meaningful target genes (Figure 4(d)).

In order to verify this screening, real-time fluorescent quantitative PCR was conducted to detect downstream genes screened in the DU145 cell line after ZFP36 overexpression and knockout. mRNA expression of all genes in DU145 cells knocked out ZFP36 elevated markedly. In DU145 cells that overexpressed ZFP36, CDK6 and TGFBR2 mRNA expression was substantially reduced, but CDK6 reduction was more significant (Figures 4(e) and 4(f)). (CDK6 mRNA expression in the ZFP36 overexpression group decreased significantly, about 0.1144 times as low as control; however, CDK6 mRNA expression increased significantly in the ZFP36 knockout group, about 14.1777 times that of the control group).

Additionally, mRNA levels of downstream genes in nude mouse-transplanted tumor tissues were also determined. The results showed that in the ZFP36 knockout group, the expression of CDK6 was approximately 16.6771 times and 27.7519 times of the control, respectively, with an evident increase (Figure 4(g)), no apparent change was revealed in CDK6 expression in the ZFP36 overexpression group (Figure 4(h)). Furthermore, CDK6 was of vital importance in both PI3K-Akt and cell cycle signaling pathways involved in differentially expressed proteins after ZFP36 inhibition. Therefore, we further verified biological roles of the ZFP36-CDK6 axis in PCa progression in our experiments.

To further illustrate the effect of ZFP36 on the level of CDK6 protein, we detected relative changes in CDK6 protein expression in the ZFP36 overexpression cell line via western blot. The expression of CDK6 protein greatly reduced in the DU145-ZFP36 group versus DU145-NC (control group) (Figure 5(a)), whereas that of CDK6 was greatly elevated in the DU145-KO-ZFP36 group (Figure 5(b)), indicating that ZFP36 could negatively mediate CDK6 protein expression.

To confirm that ZFP36 targeted CDK6, we constructed the 3′-UTR AU region of CDK6 mRNA. It contains complementary sequence of ZFP36 luciferase reporter gene (wild type). Meanwhile, the 3′-UTR AU region of CDK6 mRNA was deleted and the complementary sequence of ZFP36 (DEL type) luciferase reporter gene (Figures 5(c) and 5(d)). The determination of luciferase activity indicated a great reduction of the expression of CDK6 reporter gene following cotransfection with ZFP36 mimic. Conversely, CDK6 reporter gene changed little with sequence deletion of the same fragment after cotransfection with the ZFP36 mimic (Figure 5(e)). The results revealed that the 3′-UTR AU region ARE sequence of CDK6 mRNA was the complementary site of ZFP36, indicating that CDK6 might be a direct target of ZFP36.

We subsequently employed RNA immunoprecipitation (RIP) to further demonstrate whether there was a direct interaction between ZFP36 protein and CDK6 mRNA. In this experiment, the transfection target protein group was used as the RIP experimental group, and the transfected empty plasmid group was used as the RIP-negative control group. CDK6 was greatly enriched in the experimental group versus control, indicating an interaction between ZFP36 and CDK6 (Figures 5(f) and 5(g)). All of the described results revealed that ZFP36 mediated CDK6 expression negatively by binding to AREs of CDK6.

### 3.11. ZFP36 Regulates Prostate Cancer Cell Cycle

We have shown that ZFP36 can target and negatively regulate CDK6 expression, and CDK6 acts as an essential component of cell cycle signal regulation pathway. Therefore, we further verified whether ZFP36 overexpression and knockout affected PCa cell cycle. Compared with the NC group, DU145 cells at the S+G2 phases were significantly increased following ZFP36 knockout, and the G1 phase was significantly decreased (Figure 6(a)); on the contrary, DU145-pre-ZFP36 at the S+G2 phases were greatly decreased, but increased significantly at the G1 phase (Figure 6(b)), and both revealed significant differences. It is suggested that ZFP36 blocked the tumor cell cycle in the G1 phase, thereby inhibiting tumor growth.

### 3.12. ZFP36 Affects Cell Cycle Progression and Regulates Gene Expression in PCa Cells

In order to further clarify its potential mechanism, we tested many cell cycle-related regulators downstream of CDK6. The DU145 cell line with overexpression and knockdown of ZFP36 was constructed and verified. The cell line was identified by western blot (Figures 6(c) and 6(d)). The identification results showed that the cell construction was successful. Relevant proteins were further identified using western blot analysis, suggesting that CDK2, CDK6, cyclin D1, cyclin D2, E2F1, and c-Myc levels in DU145 cells overexpressed by ZFP36 continued to decrease, while the level of P27 was significantly elevated (Figure 6(e)). The knockout DU145 cell line showed the opposite result (Figure 6(f)). Therefore, ZFP36 prevented the growth of the G1 phase by negatively regulating CDK6 and cyclin.

### 3.13. Oxidative Stress Mediates ZFP36 Regulation in Prostate Cancer

To explore whether oxidative stress is related to ZFP36 regulation in PCa, we screened 1708 DEGs related to oxidative stress in PCa patients and used STRING to find 23 genes related to ZFP36 or CDK6. The Venn diagram presented five overlapped genes in the intersection set (Figure 7(a)). GO enrichment showed that the genes associated with response to oxidative stress are DUSP1 and FOS (Figures 7(b) and 7(c)). Importantly, DUSP1 and FOS interacted directly with ZFP36 (Figure 7(d)). Therefore, we guessed oxidative stress mediated the regulation of ZFP36 in PCa by DUSP1 or FOS.

In addition, we verified whether it was involved in the regulatory process of ZFP36 by measuring oxidative stress-related indicators in DU145 cells. Compared with control, MDA and ROS contents were significantly decreased following ZFP36 overexpression, but significantly increased in the knockout of ZFP36 (Figures 7(e) and 7(f)). The SOD enzyme activity was markedly increased in the ZFP36 overexpression group but greatly decreased after ZFP36 knockout (Figure 7(g)). Oxidative stress exerted certain effects on the regulation of PCa by ZFP36.

## 4. Discussion

It is well recognized that PCa is a heterogeneous cancer; some tumors are indeed very aggressive and can progress rapidly, while others do not develop for years or decades, ideally requiring only monitoring and no treatment. Because of this heterogeneity, it is difficult to determine which genetic abnormality contributes to prostate cancer initiation, progression, and ultimately treatment resistance [26, 27]. Therefore, in order to improve the diagnostic ability of prostate cancer, find more accurate molecular markers, and provide personalized treatment services, it has always been a hot spot in urological research. The role of RNA has been demonstrated in PCa. For example, PCa progression can be promoted by long noncoding RNA BCYRN1 through elevated HDAC11 [22–28] and by circular RNA circFOXO3 via miR-29a-3p [29]. However, there are fewer studies on ZFP36 in PCa, and this study validated the regulatory role of ZFP36 in PCa based on TCGA database and experiments.

mRNAs encode many proteins involved in tumorigenesis and progression, and their 3′-UTRs contain ARE-like sequences, and therefore, they are likely to be regulated by one or more ARE-BPs through posttranscription. Through TCGA and Taylor databases, we found that ZFP36 expression, a RNA-binding protein, links intimately to PCa biochemical recurrence, and the lower the expression of ZFP36, the lower the survival of PCa patients; the higher the degree of malignancy, and the higher occurrence of distant metastasis, and so the probability. These data suggest that ZFP36, a protein with mRNA binding and instability, is of great significance in PCa growth and tumorigenesis.

The current study determined that elevated levels of ZFP36 expression were inversely correlated with aggressive progression and limited survival time in PCa patients, and it was recognized as a novel PCa suppressor. Significantly, the findings or the present research demonstrated that ZFP36 functioned as a PCa tumor suppressor. By upregulating ZFP36 expression in PCa cells, we demonstrated that ZFP36 could impair the in vitro proliferation, migration, and invasion of PCa cells. Furthermore, ZFP36 activation hindered the use as subcutaneous xenografts in the ability to grow in the body in DU145 and 22RV1 cells. These results are consistent with those of B cell lymphoma in a mouse model driven by myc cells, where enhanced ZFP36 expression in B cells impedes lymphoma maintenance in an allograft model [16]. Interestingly, a recent study has revealed that ZFP36 can directly bind interleukin- (IL-) 23, cyclooxygenase- (COX-) 2, and VEGF in the 3′-UTRs, thereby reducing the stability and expression in colon cancer and ZFP36 depletion results in colon cancer cell proliferation [30]. As for breast cancer, ZFP36 deletion can upregulate cytokines IL-16, COX-2, and VEGF, which are intimately associated with cell proliferation [31]. ZFP36 is also predicted to be a promising upstream inhibitor of the NF-*κ*B pathway, with a role in reversing the growth of PCa [32]. Taken together, novel therapeutic approaches that specifically stimulate ZFP36 expression can be a potential way to treat tumors with low ZFP36 expression.

In addition, RNA-Seq analysis was conducted to determine whether there were biological pathways directly influenced by ZFP36 expression in PCa. Over 300 genes with changes in expression were identified due to ZFP36. Surprisingly, ZFP36-induced differentially expressed gene pathway analysis in PCa cells identified genes involved in tumorigenesis, including PI3K-Akt signaling, Rap1 signaling, circadian rhythm, cell-matrix adhesion, and HIF-1 signaling pathway, and the cancer pathway was significantly correlated. Most importantly, CDK6 was recognized as a downstream target gene of ZFP36. The cell cycle kinase CDK6 is a cell cycle-dependent kinase and transcriptional regulator. Cell cycle disorder is an important mechanism affecting tumorigenesis. During the regulation process of cell cycle, cyclin and cyclin-dependent kinase abnormalities can lead to tumorigenesis, such as Polo-like. The mRNA of protein kinase 3 consists of 3 AREs in the 3′-UTR, and ZFP36 affects cell cycles via modulating mRNA degradation. In lung cancer, ZFP36 destabilizes cyclin B1 mRNA and reduces its expression [33]. As a tumor suppressor gene, large tumor suppressor kinase 2 (LATS2) is essential for cell cycle inhibition [34]. An ARE has been identified containing in the 3′-UTR of its mRNA, so ZFP36 reduces cyclin B1 and LATS2 by reducing cyclin B1 and LATS2 expression to regulate the lung cancer cell cycle. Transcription factor C-Jun is regarded as a protooncogene of breast cancer. Being a key member of activator protein- (AP-) 1 complex, it can accelerate the cell cycle [35]. The interaction between AP-1 and c-Jun can realize induced cell cycle arrest in breast cancer. TTP has been indicated to have the ability of binding to c-Myc and cyclin D1 mRNA AREs and downregulating their expression levels in glioma [36], which can precisely regulate the glioma cell cycle.

Here, we expressed interest in whether CDK6 has a biological function as the downstream target of ZFP36, and for further validation, we found CDK6 at mRNA level and protein levels in PCa cells and tumor xenografts with enhanced and depleted ZFP36 expression decreased and increased, respectively, demonstrating the negative regulatory effect of ZFP36 on CDK6, which was further confirmed using luciferase reporter and RNA coimmunoprecipitation assays. Meanwhile, CDK6 was newly discovered as a direct target of ZFP36. It can mediate cell cycle progression at the G1 stage and transition at the G1/S stages [37]. Therefore, we also confirmed in cell cycle experiments that ZFP36 blocks tumor cell cycle in the G1 phase, thereby inhibiting tumor growth. In mammalian cells, CDK6 activates the cell cycle via several interactions with cyclins D1, D2, and D3 during early G1 [38]. As it is related to cell proliferation, CDK6 is reported to be abnormally expressed in lymphoma, medulloblastoma, leukemia, and melanoma due to chromosomal rearrangements [39, 40]. We further identified the downstream effectors of the ZFP36-CDK6 axis and found that the levels of CDK2, CDK6, cyclin D1, cyclin D2, E2F1, and c-Myc were all decreased, while the level of P27 was significantly increased in ZFP36-overexpressing DU145 cells. This data is consistent with the report of Lee et al. in prostate cancer [41], which more fully demonstrates that ZFP36 prevents tumor cell growth in the G1 phase by negatively regulating CDK6 and cyclins. Some researchers have also pointed out that CDK6 is related to the occurrence of tumors, and clinical trials of its inhibitors have shown good safety and efficacy, suggesting that CDK6 can be a promising target for cancer management, which confirms the anticancer potential of ZFP36 from the side.

A central finding of the current research is that suppressed ZFP36 expression usually occurs in human cancer, of which the functional reduction can modulate distinct tumorigenic phenotypes. Reduced expression of ZFP36 in PCa patients might be an indicator of negative prognosis, since low ZFP36 mRNA may develop more advanced tumors, increasing their risks of cancer recurrence and death. In addition, the encouraging finding of this study is that some studies have reported that average level of zinc in PCa tissues is evidently decreased compared with BPH and normal prostate, and zinc is an essential element for zinc finger protein generation; therefore, it is a bold guess that the reduction or absence of zinc may be an important reason for the decreased expression of ZFP36. The aggressive development of PCa might result from a fundamental metabolic transformation that prevents malignant cells from accumulating zinc [42]. This study presented clinical and biochemical evidence, suggesting that alterations in zinc metabolism may be of vital importance in PCa pathogenesis, and timely zinc supplementation may improve ZFP36 expression levels, thereby inhibiting prostate cancer development, which needs to be further confirmed in follow-up studies.

In addition, oxidative stress has an association with PCa [43]. Normal physiological levels of androgens can maintain the balance between ROS and antioxidant enzymes, apoptosis, and proliferation in the prostate [44]. Androgen deprivation therapy (ADT) disrupts normal androgen status by blocking androgen receptor (AR) signaling and increases mRNA levels of three reduced nicotinamide adenine dinucleotide phosphate (NADPH) oxidases in vivo, such as Nox1, Nox2 (gp91phox), and Nox4, while also decreasing the expression levels of antioxidant enzymes, namely, thioredoxin1, manganese superoxide dismutase, and glutathione peroxidase1, leading to excessive ROS production and exacerbating oxidative stress [45]. In this study, bioinformatics analysis revealed that oxidative stress may mediate the regulation of ZFP36 in PCa. Through experimental validation, it was found that after overexpression of ZFP36 in DU145 cells, MDA and ROS levels, indicators related to oxidative stress, were decreased and SOD enzyme activity was increased as measured, implying that oxidative stress can regulate PCa by ZFP36.

Although this study demonstrated a significant role of ZFP63 in PCa, some limitations are also needed to be further improved. For example, despite reduced zinc expression in human PCa tissues, we did not further elucidate the direct correlation between this result and the role of ZFP63. In addition, we only analyzed the possible role of oxidative stress in this process through bioinformatics but did not further verify it through experiments.

In conclusion, our data provide compelling evidence that strongly supports the proposal that ZFP36 acts as a potential prognostic biomarker. Deregulation of ZFP36 is responsible for cell proliferation and promotes PCa migration and invasion via regulating CDK6 signaling pathway. Meanwhile, the ZFP36-CDK6 axis which has been lately discovered elucidates the molecular mechanism of PCa progression and a novel therapeutic target of PCa therapy. Furthermore, it is exciting that supplemental intake of zinc may be another breakthrough point in ZFP36 expression. In the future, we can effectively provide new strategies and targets for PCa treatment by deeply investigating oxidative stress in regulating PCa by ZFP36 and related signaling pathways.

## Figures and Tables

**Figure 1:** (a) ZFP36 expressed higher in normal tissues than cancer tissues based on TCGA database. (b–d) ZFP36 expression in prostate cancer and normal tissues. (e, f) Correlation between ZFP36 expression and PCa patients' survival (^∗^*P* < 0.05, ^∗∗^*P* < 0.01, and ^∗∗∗^*P* < 0.001). Note: the sample messages in (b) and (c): TCGA contains 498 PCa and 52 normal tissues; Taylor contains 150 PCa and 29 normal tissues. Sample replicate value *n* = 3 in (d).

**Figure 2:** (a–d) Western blot verification of ZFP36 overexpression and knockdown models (DU145 and 22RV1). Effects of overexpression and inhibition of ZFP36 on tumor cell (e, h) proliferation (DU145 and 22RV1), (f, i) migration (DU145 and 22RV1), and (g, j) and invasion (DU145 and 22RV1). ^∗^*P* < 0.05, ^∗∗^*P* < 0.01, and ^∗∗∗^*P* < 0.001. Scar bar: 400 *μ*m in the 100x figure and 200 *μ*m in the 200x figure. *n* = 3.

**Figure 3:** (a–d) The nude mouse tumor-bearing model suggests that overexpression of ZFP36 inhibits the growth of prostate cancer xenografts. (e) Immunohistochemistry detection of related protein expression in PCa transplanted tumor tissues (^∗^*P* < 0.05, ^∗∗^*P* < 0.01). Scar bar: 50 *μ*m. Note: sample replicate values for each time point *n* = 6 in (b) and *n* = 4 in (d). Sample replicate value *n* = 3 in (e).

**Figure 4:** The related pathways of ZFP36 in prostate cancer: (a) Volcano diagram, (b) GO, and (c) KEGG pathway enrichment analysis of ZFP36-related genes. (d) Screening map of downstream genes. (e, f) Effects of ZFP36 on the downstream gene (DU145 cell line) mRNA expression and (g, h) animal transplanted tumor tissue (^∗^*P* < 0.05, ^∗∗^*P* < 0.01, and ^∗∗∗^*P* < 0.001). *n* = 3.

**Figure 5:** (a, b) Negative regulation of ZFP36 on the downstream gene CDK6. (c–e) ZFP36 targeting downstream gene CDK6. (f, g) ZFP36 targeting downstream gene CDK6. ^∗^*P* < 0.05, ^∗∗^*P* < 0.01, and ^∗∗∗^*P* < 0.001. *n* = 3. (f) Input is the total cell protein, the control group is the RIP-negative control group, the experimental group is the RIP experimental group, the picture is the WB result of the product during the RIP process, the experimental result is positive, indicating that this experiment is based on the ZFP36 protein Bait protein, and the experiment of obtaining ZFP36-RNA complex is successful. (g) The result of qPCR detection of CDK6 gene expression level of the product obtained by RIP.

**Figure 6:** (a, b) The effect of ZFP36 on prostate cancer cell cycle. (c, d) Western blot identification of DU145 cell lines. (e, f) Effects of ZFP36 on the cycle-related proteins in PCa cells (^∗^*P* < 0.05, ^∗∗^*P* < 0.01, and ^∗∗∗^*P* < 0.001). *n* = 3.

**Figure 7:** (a) Screening map of the intersection gene. (b, c) GO enrichment analysis of 5 intersection genes. (d) PPI network map. (e, f) Determination of MDA and ROS content and SOD enzyme activity by enzyme-linked immunosorbent assay (^∗∗^*P* < 0.01). *n* = 3.

**Table 1:** Zinc in normal, benign prostatic hyperplasia, and PCa tissues (reference data).

Author	Year	Methods	Zn (*μ*g/g dry tissue)					
			Normal		BPH		Prostate cancer	
			*N*	Mean	*N*	Mean	*N*	Mean
Mawson et al.	1952	SAS	7	895 ± 96 SE	20	772 ± 93 SE	5	190 ± 61 SE
Hoare et al.	1956	SAS	19	744 ± 124 SE	52	486 ± 26 SE	18	273 ± 52 SE
Shirakawa et al.	1961	—	—	790	—	751	—	390
Schrodt et al.	1964	XRF	—	540 ± 100 SE	9	1902 ± 395 SE	10	282 ± 32 SE
GyOrkey et al.	1967	AAS	10	1055 ± 420	10	3800 ± 65 SD	10	230 ± 6 SD
Hienzsch et al.	1970	AAS	60	438	34	855	4	78
GyOrkey et al.	1973	AAS	3	263 ± 15 SE	8	607 ± 45 SE	3	80 ± 7 SE
Mukhitdinov et al.	1975	AES	82	107 ± 14 SE	61	215 ± 5 SE	4	147 ± 11 SE
Wallace et al.	1975	AES	—	—	13	1210 ± 901 SD	3	432 ± 238 SD
Habib et al.	1976	AAS	9	447 ± 79 SE	23	452 ± 78 SE	9	171 ± 29 SE
Dunchik et al.	1977	XRF	11	1330 ± 156 SE	18	1467 ± 539 SE	23	442 ± 58 SE
Jafa et al.	1980	AAS	10	2734 ± 12 SE	10	3770 ± 13 SE	10	814 ± 17 SE
Feustel et al.	1982	AAS	16	348 ± 269 SD	24	774 ± 524 SD	36	147 ± 103 SD
Marezyfiska et al.	1983	AAS	8	965 ± 435 SD	43	851 ± 410 SD	12	320 ± 147 SD
Lahtonen et al.	1985	AAS	—	—	15	904 ± 111 SE	3	160 ± 57 SE
Feustel et al.	1987	AAS	5	488 ± 190 SD	10	1177 ± 485 SD	9	413
Zaichick et al.	1997	XRF	37	1018 ± 124 SE	50	1142 ± 77 SE	59	146 ± 10 SE
Pamela et al.	2011	AAS	20	1009 ± 155 SD	45	387 ± 86.1 SD	18	175 ± 58.6 SD

AES: atomic emission spectrometry; SAS: solution absorption spectrometry; XRF: X-ray fluorescent spectrometry; AAS: atomic absorption spectrometry; SD: standard deviation; SE: standard error of the mean.

**Table 2:** Correlation between ZFP36 mRNA expression and clinical characteristics of PCa patients.

Clinical characteristics	ZFP36 expression in TCGA dataset			ZFP36 expression in Taylor dataset		
	Cases	Mean ± SD	*P* value	Cases	Mean ± SD	*P* value
*ZFP36 expression*						
Benign	52	13.04 ± 1.35	0.012	29	9.03 ± 0.76	0.024
Cancer	498	12.49 ± 1.52		150	9.47 ± 0.97	
*Age (years)*						
<60	201	12.47 ± 1.45	0.839	93	9.55 ± 0.92	0.157
≥60	296	12.50 ± 1.55		57	9.32 ± 1.05	
*Serum PSA (ng/mL)*						
<4	—	—	—	24	9.78 ± 0.92	0.091
≥4	—	—		123	9.41 ± 0.98	
*Gleason scores*						
<8	292	12.66 ± 1.49	0.002	117	9.72 ± 0.86	<0.001
≥8	206	12.24 ± 1.52		22	8.74 ± 0.84	
*Clinical stage*						
<T2A	177	12.60 ± 1.49	0.073	80	9.44 ± 0.96	0.261
≥T2A	229	12.34 ± 1.44		65	9.61 ± 0.93	
*Pathological stage*						
<T3A	186	12.73 ± 1.48	0.002	86	9.70 ± 0.90	0.016
≥T3A	304	12.31 ± 1.48		55	9.31 ± 0.96	
*Metastasis*						
No	416	12.53 ± 1.51	0.143	122	9.66 ± 0.87	<0.001
Yes	82	12.27 ± 1.56		28	8.61 ± 0.96	
*Overall survival*						
Alive	487	12.49 ± 1.51	0.599	131	9.57 ± 0.93	<0.001
Die	10	12.23 ± 1.45		19	8.74 ± 1.02	
*PSA failure*						
Negative	439	12.56 ± 1.51	0.003	104	9.74 ± 0.88	<0.001
Positive	59	11.95 ± 1.46		36	9.01 ± 0.89	
*Surgical margin status*						
Negative	314	12.52 ± 1.52	0.727	—	—	—
Positive	153	12.47 ± 1.49		—	—	

**Table 3:** Correlation between clinicopathological characteristics and biochemical recurrence-free survival of PCa patients.

Parameters	Univariate analysis		Multivariate analysis	
	HR (95% CI)	*P*	HR (95% CI)	*P*
ZFP36	0.764 (0.630-0.926)	0.006	0.767 (0.625-0.942)	0.012
Age	1.019 (0.979-1.061)	0.351	1.012 (0.969-1.057)	0.580
Gleason score	2.074 (1.583-2.717)	<0.001	1.842 (1.320-2.572)	<0.001
Pathological stage (T2 vs. T3)	5.110 (2.189-11.928)	<0.001	2.145 (0.839-5.481)	0.111
Clinical stage (<T2A vs. ≥T2A)	3.378 (1.688-6.759)	0.001	2.284 (1.112-4.692)	0.025
Surgical margin (+ vs −)	1.856 (1.087-3.166)	0.023	1.044 (0.554-1.970)	0.893

Note: HR: hazard ratio; CI: confidence interval.

## Data Availability

All data, models, and code generated or used during the study appear in the submitted article.
